RETRACTED

# Cisapride versus Maren Pill for Functional Constipation: A Meta-Analysis

**DOI:** 10.1155/2022/7619998

**Published:** 2022-05-12

**Authors:** Yanming Sun, Ying Zhu, Rui Ye

**Affiliations:** Critical Care Medicine, Affiliated Hangzhou First People's Hospital, Zhejiang University School of Medicine, Hangzhou, Zhejiang, China

## Abstract

**Background:**

The efficacy and safety of cisapride in functional constipation (FC) remain unclear. This meta-analysis aimed at investigating the efficacy and safety of cisapride and Maren pill in the treatment of FC. *Material and Methods*. PubMed, Web of Science, Embase, Cochrane Library, WANFANG DATA, VIP, and CNKI databases were searched from inception to December 2021 for eligible comparative studies investigating the effects and safety of cisapride and Maren pill for FC. The primary outcome was the therapeutic effectiveness rate. The secondary outcomes were recurrence rate and incidence of adverse events.

**Results:**

A total of 526 studies were screened out by searching the electronic databases and by manually searching the relevant reference lists. According to the four-step process (identification, screening, eligibility, and inclusion) to select studies for meta-analysis, 521 articles were excluded. Finally, 5 studies with a total of 414 patients with FC were included in the quantitative analysis after sequential exclusion. The cisapride group had a significantly higher effectiveness rate than the control one (90.78% vs 64.97%, *P* < 0.05). The incidence of adverse events in the cisapride group was lower than that in the Maren pill group (10.08% vs 13.95%, *P* < 0.05). Similarly, the recurrence rate of the cisapride group was lower than that of the Maren pill group (32.31% vs 53.16%, *P* < 0.05).

**Conclusion:**

For FC patients, cisapride is more effective than Maren pill; the recurrence rate and adverse event rate are lower than the latter, which makes it a better choice. The combination of cisapride and Maren pill is a direction of future research studies, which may increase the efficiency and reduce the dosage of cisapride.

## 1. Introduction

Constipation is a series of syndromes with reduced number of bowel movements and defecation difficulty [1]. Due to the changes in modern diet, the increase of work stress, and the change of life environment, the prevalence of constipation has increased gradually [2, 3]. It seriously affects people's quality of life and increases the risk of cardiovascular and cerebrovascular diseases, digestive tract tumors, Alzheimer's disease, and hepatic encephalopathy. Functional constipation (FC) is a common cause of chronic constipation. Several studies have shown that functional diseases are the most common causes of constipation in chronic constipation, accounting for 57.1% [4]. The side effects of common laxatives are serious. Long-term use of laxatives such as castor oil, rhubarb, and phenolphthalein can degenerate the intestinal myenteric plexus, making constipation more stubborn, and may cause colonic and intestinal black lesions [5]. Recent studies have found that most patients have intestinal dysmotility.

RETRACTED

Cisapride belongs to benzamide derivatives and is a novel all-gastrointestinal motility drug. It facilitates acetylcholine release from the enteric cholinergic neurons through a selective 5-hydroxytryptamine (5-HT, serotonin) 4 receptor agonistic action [6]. It has been used in treating upper-GT disorders such as abdominal discomfort, nausea, and vomiting that are caused by delayed gastric emptying due to diabetes, gastroesophageal reﬂux disease, and nonulcer dyspepsia [7].

However, the efficacy and adverse events of cisapride in improving symptoms of FC still remain controversial. Furthermore, there is no systematic meta-analysis to evaluate the efficacy and safety of cisapride in patients with FC. The aim is to perform a systematic meta-analysis to evaluate the efficacy and safety of cisapride in the treatment of FC by integrating existing controlled studies.

## 2. Methods

### 2.1. Literature Search

We conducted a literature search without a language restriction to identify relevant available articles that had been published within the databases from their inception to December 2021. Relevant studies and systematic reviews were also scanned for additional eligible trials. The search terms included “functional constipation,” “Maren,” and “Cisapride.” Manual searches were also performed to identify relevant articles from the reference lists.

### 2.2. Inclusion and Exclusion Criteria

The inclusion criteria were as follows: (1) original studies on FC and (2) studies that comply with the diagnosis of chronic constipation in the International Functional Diseases (FGIDS)-Rome IV in 2016. The exclusion criteria were as follows: (1) primary and secondary digestive systemic diseases; (2) secondary constipation (identify the cause) and drug constipation; (3) acute surgical disease or surgery in the last 30 days; (4) serious merger diseases or malignancies such as cardiovascular and cerebrovascular, liver, kidney, respiratory, and hematopoietic systems; (5) severe psychological disorders or insomnia; and (6) reviews, case reports, conference abstracts, or case series.

Two investigators searched and independently reviewed all identified studies. If the two investigators were not able to reach a consensus about the eligibility of an article, the dispute was resolved through discussions with a third reviewer.

RETRACTED

### 2.3. Data Extraction and Quality Assessment

Two independent researchers systematically read the title and abstract of each study, read the full text of those studies that met the inclusion criteria, and conducted data extraction and a detailed analysis of the extracted data. The data included authors, publication year, gender, age, duration, follow-up, sample, treatment outcome, adverse events, recurrence, etc. The effectiveness was defined as the significant remission of the disease. The effectiveness was set as the primary outcome of the present study. Two authors assessed the qualities of the studies individually by using the Newcastle–Ottawa Scale (NOS). The total scores of NOS ranged from 0 to 9 and were categorized into three groups.

### 2.4. Statistical Analysis

Dichotomous data were reported as odds ratios with their 95% confidence intervals (CIs). The mean difference and the 95% CI were calculated for the continuous variable. Publication bias was evaluated by a funnel plot. *P* values <0.05 were considered to be statistically signiﬁcant in all analyses. Heterogeneity was assessed by the chi-squared test and quantified using the *I*^2^ statistic. If *P* > 0.10 and *I*^2^ < 50%, the heterogeneity was acceptable and a ﬁxed-effect model would be used for data analysis. If *P* > 0.10 or *I*^2^ ≥ 50%, we would search the reasons of heterogeneity and use a random-effects model. The Revman was used for the meta-analysis in the present study.

## 3. Results

### 3.1. Characteristics of the Included Studies

A total of 526 studies were screened out by searching the electronic databases and by manually searching the relevant reference lists. According to the four-step process (identification, screening, eligibility, and inclusion) to select studies for meta-analysis, 521 articles were excluded. Finally, 5 studies with a total of 414 patients with FC were included in the quantitative analysis after sequential exclusion (Figure 1).  Table 1 shows the characteristics of the studies [8–12]. The NOS scores of all the included studies were 7 or 8, which indicated that they had a low risk of bias. The mean age of the patients with FC was 39 to 65 years, and the male-to-female ratio was approximately 236 to 178 within the included studies.

### 3.2. Effective Rate

As shown in Figure 2, we compared cisapride and Maren pill in terms of their effective rates. In the cisapride group, 197 were deemed effective and the effective rate was 90.78% (197/217); in the Maren pill group, the number of patients who received effective treatments was 128 and the effective rate was 64.97% (128/197). The effective rate of the cisapride group was significantly higher than that of the Maren pill group. The heterogeneity test results showed that *P* *=* *0.89* and *I*^2^ *=* *0%*, indicating there was no significant heterogeneity in the included studies. And, a fixed-effect model was used. For evaluation of publication bias, the funnel plot (Figure 3) showed no significant publication bias between the included studies in the analyses.

RETRACTED

### 3.3. Recurrence Rate

We compared the recurrence rate between the two groups. The data are presented in Table 2. The recurrence rate was the ratio of the number of relapses to the number of actives. Two studies lacked relevant data. Based on the statistics of the remaining 3 studies, the total number of relapses was 63 and the total recurrence rate was 32.31% (63/195). In the cisapride group, 21 patients had recurred and the recurrence rate was 18.10% (21/116). In the Maren pill group, 42 patients had recurred and the recurrence rate was 53.16% (42/79). The difference in the recurrence rate between the two groups was statistically significant; the recurrence rate in the cisapride group was lower than that in the Maren pill group.

### 3.4. Adverse Events

Table 3 shows the adverse events. The total number of adverse events was 26, including 3 types: 17 cases of abdominal pain, 3 cases in the cisapride group and 14 cases in the Maren pill group; 4 cases of vomiting, 2 cases in the cisapride group and 2 cases in the Maren pill group; 5 cases of loose stool, 3 in the cisapride group and 2 cases in the Maren pill group. The total number of adverse events was 26, accounting for 10.08% (26/258). In the cisapride group, 8 patients had adverse events, accounting for 6.20% (8/129); in the Maren pill group, 18 patients had adverse events, accounting for 13.95% (18/129). The difference in the incidence of adverse events between the two groups was statistically significant, and the incidence of adverse events in the cisapride group was lower than that in the Maren pill group (Table 4).

## 4. Discussion

In recent years, the prevalence rate of FC has gradually increased, which has generated a serious negative impact on patients' daily lives and work. Several studies have shown that FC could lead to a variety of complications and aggravate or cause rectal and anal diseases, which may trigger neurogenic or systemic diseases, so it is very important to implement effective treatment. [13].

Maren pill could effectively shorten the interval of bowel movements, improve the quality of life, and alleviate the psychological problems of patients. And, it could be used for long-term constipation in the elderly, constipation after surgery, and constipation caused by opioids, with a low probability of adverse events [14, 15]. Several studies reported that it could be used to improve the constipation symptoms and nutritional status of patients with acute exacerbation of chronic obstructive pulmonary disease and sepsis. It can effectively alleviate the constipation problems of stroke patients. The effect on constipation caused by antipsychotic drugs was significant [16].

RETRACTED

Cisapride is a substituted benzamide compound that stimulates motor activity in all segments of the gastrointestinal tract by enhancing the release of acetylcholine from the enteric nervous system [17, 18]. Cisapride is administered orally in the treatment of gastro-oesophageal reflux disease, functional dyspepsia, gastroparesis, chronic intestinal pseudo-obstruction syndromes, and chronic constipation. Cisapride in combination with MgO may have a synergistic effect and improve the frequency of stool passage in pediatric FC. However, several studies suggested that cisapride could not be reasonably used in chronic constipation or irritable bowel disease [19–21]. Its effectiveness and safety were questioned mainly due to its serious adverse events. Here, we assessed systematically the efficacy and safety of cisapride in relieving constipation. Additionally, the sample size in the present meta-analysis was not large, which might lead to bias.

## 5. Conclusion

Compared to Maren pill, cisapride is more effective with lower recurrence rate and lower incidence of adverse events in the present study. For patients with simple FC, cisapride is an effective drug with rapid onset, low recurrence rate, and few complications. Cisapride is one of the common gastrointestinal motility drugs and is a highly selective 5-HT4 receptor antagonist for intestinal motility. Considering the severe fatal complications of the heart system, it is more suitable for short-term treatment. Maren pill has a slightly slower onset, and patients need to be treated for a longer time. Therefore, it is easy to be low when calculating the efficiency, and the recurrence rate is high for patients taking short-term medication. In addition, the patients included in this study were FC patients without other complications. There are no obvious complications in this study, and cisapride is safe and effective for people without other diseases. On the other hand, Maren pill is a Chinese patent medicine with laxative effect. It is more suitable for long-term treatment of chronic constipation and patients with complications, and further research studies are needed. Finally, the combination of cisapride and Maren pill is a direction of future research studies, which may increase the efficiency and reduce the dosage of cisapride.

RETRACTED

## Figures and Tables

**Figure 1:** Identification of studies for inclusion.

**Figure 2:** Forest plot of effective rate.

**Figure 3:** Funnel plot of effective rate.

**Table 1:** Basic characteristics of the included studies.

First author	Publication year	Group (n)	Patients age, years	Sex (M : F)	Duration, months	Effective	Ineffective	Adverse events	Recurrence	NOS
He et al.	2010	Cisapride (50)	21～63	24 : 26	>12	43	7	3	10	7
		Maren (50)	22～65	29 : 21	>12	23	27	0	13	

Liu et al.	2017	Cisapride (48)	64.5 ± 6.5	29 : 19	NA	45	3	NA	NA	8
		Maren (48)	64.1 ± 7.3	27 : 21	NA	34	14	NA	NA	

Shi et al.	2003	Cisapride (40)	18～74	25 : 15	NA	36	4	NA	NA	7
		Maren (20)	19～70	10 : 10	NA	15	5	NA	NA	

Yang et al.	2017	Cisapride (49)	50.21 ± 1.17	29 : 20	NA	45	4	3	5	8
		Maren (49)	51.45 ± 1.25	28 : 21	NA	35	14	10	15	

Zhang et al.	2019	Cisapride (30)	38.75 ± 5.73	17 : 13	6.35 ± 2.61	28	2	2	6	8
		Maren (30)	38.69 ± 5.68	18 : 12	6.42 ± 2.58	21	9	8	14	

Notes: *M*, male; F, female; NA, not available; age: mean ± standard deviation (SD) or range; NOS: Newcastle–Ottawa Scale.

**Table 2:** The comparison of recurrence rate.

Studies	Cisapride group		Maren pill group		*χ* ^2^	*P*
	Yes	No	Yes	No		
He 2010	10	33	13	10	26.41	0.001
Yang 2017	5	40	15	20		
Zhang 2019	6	22	14	7		

**Table 3:** Details of adverse events in the enrolled studies.

Studies	Groups	Adverse events		
		Abdominal pain	Vomiting	Loose stools
He 2010	Cisapride	1	1	0
	Maren pill	7	1	0

Yang 2017	Cisapride	1	0	2
	Maren pill	0	0	0

Zhang 2019	Cisapride	1	1	1
	Maren pill	7	1	2

**Table 4:** The statistics of adverse events.

Studies	Cisapride group		Maren pill group		*χ* ^2^	*P*
	Yes	No	Yes	No		
He 2010	3	47	0	50	4.277	0.039
Yang 2017	3	46	10	39		
Zhang 2019	2	28	8	22		

## Data Availability

The data used to support this study are available on request.
